# Chemistry and Biology of Essential Oils of Genus *Boswellia*

This article has been retracted.

**DOI:** 10.1155/2013/140509

**Published:** 2013-03-06

**Authors:** Hidayat Hussain, Ahmed Al-Harrasi, Ahmed Al-Rawahi, Javid Hussain

**Affiliations:** ^1^Department of Biological Sciences and Chemistry, College of Arts and Sciences, University of Nizwa, Birkat Al-Mouz, 616 Nizwa, Oman; ^2^Department of Chemistry, University of Paderborn, Warburger Straße 100, 33098 Paderborn, Germany

## Abstract

The properties of *Boswellia* plants have been exploited for millennia in the traditional medicines of Africa, China, and especially in the Indian Ayurveda. In Western countries, the advent of synthetic drugs has obscured the pharmaceutical use of *Boswellia*, until it was reported that an ethanolic extract exerts anti-inflammatory and antiarthritic effects. Frankincense was commonly used for medicinal purposes. This paper aims to provide an overview of current knowledge of the volatile constituents of frankincense, with explicit consideration concerning the diverse *Boswellia* species. Altogether, more than 340 volatiles in *Boswellia* have been reported in the literature. In particular, a broad diversity has been found in the qualitative and quantitative composition of the volatiles with respect to different varieties of *Boswellia*. A detailed discussion of the various biological activities of *Boswellia* frankincense is also presented.

## 1. Introduction

The genus *Boswellia* has approximately 20 species occurring in the dry regions spanning from west Africa to Arabia and south to the northeast region of Tanzania. In addition, its species have been found in India and Madagascar. The genus is centered in northeast Africa, where approximately 75% of the species are endemic to the area. Members of this genus are trees or shrubs that are described as having outer barks that peel in parchment flakes, a greenish inner bark, watery aromatic resins, and wood with a milky latex [1]. 

Frankincense, or olibanum, is the oleogum resin that is harvested from several different trees belonging to the genus *Boswellia*. The word frankincense is derived from the ancient French name “frankincense,” meaning “pure incense.” Frankincense is also known in Arabic as “luban,” which means “white” or “cream;” in Greek as “libanos;” in Ethiopia as “etan” [2–8]. Olibanum (frankincense) has been used as incense since ancient times [9, 10]. In recent years, it has been important in the preparation of cosmetics and perfumes. In addition, olibanum has anti-inflammatory, sedative, anti-hyperlipidemic, and antibacterial activities in Unani (Islamic) and Chinese traditional medicines [9–15].

For at least 5000 years, olibanum has been an important trade material for the civilizations located in North Africa and the Arabian Peninsula. It was a precious commercial material even before Christian times because of the interest in this incense material of the old kings and queens, such as the Queen of Saba in 700 B.C. With the dawn of Christianity, it was mentioned in the Bible as one of the presents in which the three wise men had brought to Jesus on the night he was born [16]. The wide use of this resin in religious ceremonies as incense material is still important in the Roman Catholic, Episcopal, and eastern Orthodox churches. Therefore, both the production and export of olibanum is an economic priority for countries like Somalia, Ethiopia, Oman, South Arabia, and India. Olibanum has been utilized as an important fixative in perfumes, soaps, creams, lotions, and detergents in the leading products of the perfume and cosmetic industry, as it has an oriental note in its scent. The interest of pharmaceutical companies created a third market for olibanum. Since ancient times, it has been used in folk medicine for its antiseptic, antiarthritic, and anti-inflammatory effects. For this reason, olibanum has gained increasing attention from scientists in the last 20 years to better define its medical effects and identify the constituents that are responsible for these effects [16].

## 2. Volatile Constituents of *Boswellia*

Investigations of the resin and essences or extracts of *Boswellia*, with regard to the specific volatile constituents, were reported in a series of studies [16–35] (Table 1). The chemical characterization procedures enabled a total of 340 volatiles to be identified. Due to the resin nature of frankincense, it is not surprising that the major part of the constituent volatiles belonged to the terpene and sesquiterpene families or their terpenoid derivatives (Table 1). The common compounds included *α*- and *β*-pinene, limonene, myrcene, linalool, and several others. Additionally, a series of purely hydrocarbon-terpene compounds was found. More than 30 compounds from the sesquiterpene and diterpene fractions have been identified, for example, *α*-cubebene, *γ*-cadinene, *β*-bourbonene, and *α*-phellandrene dimer, which was first reported by Basar [16]. Several oxygenated isoprenoid derivatives have also been identified, such as carbonyl derivatives (e.g., carvone, fenchone) and alcohol-containing terpene and sesquiterpene derivatives (e.g., *trans*-pinocarveol, *cis*-verbenol, and cembrenol), as well as ester-containing compounds (e.g., *α*-terpinyl acetate and bornyl acetate). In addition to these isoprenoid-derived compounds, a series of straight-chain alkyl-esters, such as octyl acetate and alcohols (decanol, hexanol), have been detected. Analyzing *B. serrata* by hydrodistillation, Singh et al. [22], Verghese et al. [23], and Camarda et al. [24] each found *α*-thujene to be the dominant substance. However, the specific values were in the range 22.7–61.4%. Although, Basar [16] claimed that myrcene was the prevalent volatile (38%), followed by *α*-thujene (12%). *α*-Pinene was found in all samples, with the relative amounts in the range of 3.3–11.2%. In the hydrodistillate of *B. carter *and *B. sacra*, the values of the detected substances differed to a major extent. Basar [16] claimed that octyl acetate (39.9%) was the main constituent, followed by 1-octanol (11.9%). Al-Harrasi and Al-saidi [25] found limonene (33.5%) and (*E*)-*β*-ocimene (32.2%) to be the predominant compounds, whereas Marongiu et al. [26] claimed that octanol acetate was the main volatile (45.2%), followed by phyllocladene (13.2%) and incensole acetate (13%). Mikhaeil et al. [20] identified duva-3,9,13-trien-1,5a-diol-1-acetate as the main volatile (21.4%), followed by octyl acetate (13.4%). Like Al-Harrasi, Camarda et al. [24] also reported limonene to be the dominant substance, albeit at half the abundance found by Al-Harrasi (18.2%). Furthermore, Camarda identified *α*-pinene as the second most abundant substance (15.1%). However, this finding is in contrast to other studies, in which the *α*-pinene contents were reported in the range of 0.7–15.1%. Baser et al. [27], Basar [16], and Camarda et al. [24] all claimed that limonene was the main constituent of *B. rivae*, with values in the range of 14.8–28.0%. Again, another dominant substance seemed to be *α*-pinene, with relative values of 5.3–16.7%. In agreement with this, *α*-pinene, together with *α*-thujene, was found as the dominant substance in *B. neglecta*, whereas the most abundant volatile in *B. papyrifera* was octyl acetate at 63.5% [24] and 56% [36]. Furthermore, Basar [16] found that *trans*-verbenol was the main volatile (15.5%) in *B. pirottae* and *α*-pinene (38%) in *B. frereana*. Summarizing the data from the analyses of the hydrodistillation extracts, *α*-pinene, limonene, octyl acetate, a-thujene, and (*E*)-*β*-ocimene can be regarded as those compounds that have been most frequently reported to be the dominant volatile constituents of the frankincense distillate. Nevertheless, these results do not allow for chemosensory interpretation of their odor contribution to the characteristic frankincense smell. In accordance with the results of the hydrodistillation, Hamm et al. [18] found *α*-thujene (with a value of 11.7%) to be the dominant volatile in a *B. serrata* extract obtained by SPME. In Basar's study [16], thujene was also mentioned, but no quantitative data was provided. For the SPME analyses, Basar reported only qualitative data and no quantitative data. Hamm reported *α*-pinene, limonene, and *β*-caryophyllene to be the main constituents in *B. carteri* and *B. sacra*. By comparison, the *α*-phellandrene dimer was the dominant volatile (20.2%) in *B. frereana*, followed by *α*-pinene (12.4%). Octyl acetate was found in the greatest abundance (64.6%) in *B. papyrifera*, followed by octanol (13.9%) [1].

Al-Saidi et al. [34] reported the volatile chemical profile and physicochemical characteristics of four commercial grades of botanically certified oleogum resins of *B. sacra*, known as Hoojri, Najdi, Shathari, and Shaabi, were studied. The striking feature of Al-Saidi et al. [34] study was the presence of high amounts of *α*-pinene in all four oils, which can be considered as a chemotaxonomical marker that confirms the botanical and geographical source of the resins. Even though many *Boswellia* species produce frankincense, the major sources of commercial frankincense are *B. serrata* (India), *B. sacra* (Oman), and *B. carteri* (Somalia). The reports on the oil composition of *B. serrata* revealed a wide variation of major constituents, but none of the studies reported *α*-pinene as the most abundant component. Similarly, reports on the oil composition of *B. carteri* from Somalia also showed variation within the major constituents, suggesting a possible existence of different chemotypes. The Al-Saidi et al. [34] study reveals that the composition pattern of three of the Omani luban oils, that is, the Hoojri, Shathari, and Shaabi oils, was different from the above cited studies in terms of the major constituent *α*-pinene. The Najdi oil, however, showed some similarity with the Somalian *B. carteri* sample studied by Abdel Wahab et al. [37], with *α*-pinene and limonene as the major constituents. The variation observed might be expected, based on several factors such as climatic changes, harvest conditions, and geographical source.

Since the entire history of *Boswellia* nomenclature is fraught with misidentification, Woolley et al. [35] showed that the history of inaccurate frankincense taxonomy also applies to the widespread error of identifying *B. carterii* as being synonymous with *B. sacra*. Woolley et al. [35] studied the essential oil of *B. carterii* and *B. sacra* and showed that *B. carterii* can always be identified by the key markers viridiflorol, cembrenol, dimethyl ethermorcinol, and most importantly incensole. *B. sacra* was distinguished by higher quantities of *α*-pinene and delta-3-carene, while *B. carterii* possessed higher quantities of *α*-thujene, myrcene, limonene, *trans*-*β*-caryophyllene, germacrene D, and incensole. Woolley et al. [35] hypothesize that the differences in enantiomeric pair ratios of monoterpenes in Arabian *B. sacra* and African *B. carterii* resins were due to the differences in the abundance of genetically expressed chiral-specific enzymes for monoterpene biosynthesis. The most likely cause of genetic shift and speciation of *B. sacra* trees in Arabia and *B. carterii* trees in East Africa was the geological isolation created by the Red Sea Rift Valley that has separated these two tectonic plate land masses. Genetic mapping of these species might provide conclusive data to support Woolley et al. observations. Woolley et al. concluded that *B. sacra* and *B. carterii* are different species based on enantiomeric pair ratios and optical rotation.

Although *α*-pinene was the major compound and found in high concentrations in all grades of Omani frankincense (*B. sacra*) [34], this compound cannot be considered as a chemotaxonomic marker for *B. sacra* because of its frequent occurrence in other species of *Boswellia* (Table 2). Frankincense is a natural oleo-gum resin whose ingredients may depend on many factors, such as location, climate, time of harvest, and other environmental conditions. An indication of this variance could be clearly seen when comparing the different results of the samples of the same species (Table 2). A remarkable diversity of the predominant compounds in similar *Boswellia* species reported by different authors is clearly seen in Table 2. For example myrcene and *α*-thujene were individually reported to be major compounds for *B. serrata*. Mikhaeil et al. [20] reported duva-3,9,13-triene-1a-ol-5,8-oxide-1-acetate to be a major compound in the essential oil of *B. carteri *whereas Basar [16] found octyl acetate to be a major compound for the same species. Limonene, *α*-pinene, and octanol were reported individually to be major constituents for *B. rivae. *The incompatibility between the results mentioned in different literature could still be logical due to the influence of several factors mentioned earlier such as the climate, harvest conditions, and geographical source. However, such contradicting results make it difficult to rely on the chemical profile of the oil as a chemotaxonomic marker to distinguish between the different commercial varieties of frankincense.

## 3. Biological Activities of Essential Oils

### 3.1. Antioxidant Activity

Awadh Ali et al. [29] evaluated essential oils of *Boswellia* species for antioxidant activity. The essential oils were able to reduce the stable free radical DPPH with IC_50_ values of 121.4 *μ*g/mL, 211.2 *μ*g/mL, and 175.2 *μ*g/mL for *B. socotrana*, *B. elongate*, and *B. ameero*, respectively. The positive factor for *B. socotrana* essential oils was the higher concentration of oxygenated monoterpenes [38, 39], but there are no data on the antioxidant activity of the oxygenated monoterpene (*E*)-2,3-epoxycarene, which is the main constituent in this oil. *Boswellia* essential oils showed lower free radical scavenging activity in comparison to other reported essential oils rich in oxygenated monoterpenes, such as *Melissa officinalis* and *M. piperita* with IC_50_ = 7.58 and 2.53 *μ*g/mL, respectively [40, 41].

Recently, Mothana et al. [31] also evaluated the antioxidant activity of essential oils of *Boswellia,* demonstrating only weak antioxidant abilities in the reduction of DPPH. The three essential oils of *B. dioscorides*, *B. elongate*, and *B. socotrana* exhibited weak radical scavenging effects (22%, 21%, and 28%, resp.) at a concentration of 1 mg/mL. In comparison, ascorbic acid had a 96% antioxidant effect. This observation was certainly associated with the low content of phenolic components, such as thymol and carvacrol, in the three investigated oils [39]. 

### 3.2. Acetylcholinesterase Inhibition

Awadh Ali et al. [29] also evaluated the AChE inhibition of essential oils of *Boswellia* species. At a concentration of 200 *μ*g/mL, essential oils of *B. socotrana* (59.3% inhibition) exhibited higher AChE inhibition than the essential oils of *B. elongata* and *B. ameero* (29.6 and 41.5% inhibition, resp.). The AChE inhibitory activity of *B. socotrana* oil may be due to the presence of (*E*)-2,3-epoxycarene and *p*-menth-1(7)-en-2-one, which belong to a group of monoterpenoid skeletons reported to have AChE inhibitory activity [42, 43]. Pulegone, a monoterpene with a *p*-menthane skeleton in *Mentha* spp, showed AChE inhibition with an IC_50_ of 890 *μ*M [42].

### 3.3. Antimicrobial Activity

Camarda et al. [24] investigated the antimicrobial efficacy of *B. carteri* against *Escherichia coli*, *Pseudomonas aeruginosa*, and three strains of *Staphylococcus aureus*. Inhibitory activity was found against all pathogens, with the highest sensitivity noted for *P. aeruginosa* at concentrations as low as 6.6 *μ*g/mL. Conversely, the essential oil of *B. carterii* was investigated for inhibitory activity against a Methicillin-resistant *Staphylococcus aureus* (MRSA) strain using a disc diffusion assay and found to have no inhibitory activity. In addition, Van et al. [32] reported that different fractions of essential oils of *B. carteri*, *B. neglecta*, *B. sacra*, *B. thurifera*, and *B. frereana* showed moderate to poor activity against a reference *S. aureus* strain (ATCC 12600). 

Mothana et al. [31] evaluated the antimicrobial activity of *B. dioscorides*, *B. elongate*, and *B. socotrana* oils against two Gram-positive bacteria, two Gram-negative bacteria, and one fungal strain. The results indicated that the oils had varying degrees of growth inhibition against the bacterial strains. However, no activity was registered against the fungus *Candida albicans*. The Gram-positive strains showed more susceptibility to the tested essential oils than the Gram-negative ones. The essential oil of *B. socotrana* demonstrated the strongest activity with the lowest MIC values (1.87 mg/mL) obtained against *Staphylococcus aureus* and *Bacillus subtilis*. 

Another study by Camarda et al. [24] demonstrated that the essential oils of four *Boswellia* species exhibited significant antifungal activity against both *Candida albicans* and *Candida tropicalis*. Camarda et al. [24] and Shao et al. [43] reported that limonene present in the essential oils was the component responsible for the antifungal activity. Hence, the absence of limonene in the essential oils explored by Mothana et al. [31] explained the lack of antifungal activity. 

The MIC values of the tested essential oils were relatively lower than those of the positive controls (3.5–7.0 lg/mL). However, as crude oils, the overall antimicrobial activity screening results were still indicative of the potential of these herbal drugs to be effective treatments for bacterial infections. Moreover, oxygenated monoterpenes, such as camphor, borneol, linalool, and *α*-terpineol, were reported to be responsible for the antimicrobial activity of several essential oils [44, 45]. Consequently, the high antibacterial efficacy of *B. socotrana* could be attributed to the high percentage of oxygenated monoterpenes, such as camphor, *α*-fenchol, terpinen-4-ol, and borneol. Moreover, the predominance of 2-hydroxy-5-methoxy-acetophenone (16.3%) could have contributed to the strong activity [31]. 

Furthermore, *B. rivae* resin essential oil was tested for its antifungal activity against *Candida albicans* ATCC 10231. In previous reports, *B. rivae* essential oils showed the lowest MIC value of 2.6 *μ*g/mL (0.3% v/v) against the same strain of *C. albicans* [24] among the oils tested. As hyphal formation is a morphogenetic process that contributes to the virulence of *C. albicans* [46], Schillaci et al. [47] opted to test the oil anti-germ tube formation activity. In this case, *B. rivae* oil demonstrated a particularly good activity as an inhibitor of germ tube formation with an IC_50_ value of 0.12 *μ*g/mL (0.014% v/v). Thus, such low IC_50_ values for *B. rivae* were a good indication that this oil also had demonstrable antibiofilm activity. In fact, the authors observed the prevention of adhesion and biofilm formation at a sub-MIC concentration of 0.88 *μ*g/mL (0.1% v/v). Moreover, the oil was significantly active at a concentration of 44.1 *μ*g/mL (5% v/v) against a preformed 24 h old *C. albicans* biofilm [47]. The chief chemical component of *B. rivae* oleogum resin oil was limonene (28%), a monoterpene hydrocarbon with demonstrated antifungal activity [48]. However, it is difficult to attribute the anti-biofilm activity to one single component, and further studies are needed to understand the role of the components of such oil in the biological activity.

Al-Saidi et al. [34] reported antibacterial activity of oleo-gum resins of *B. sacra*, known as Hoojri, Najdi, Shathari, and Shaabi against. All the four oils were effective against both Gram-positive and Gram-negative bacteria. The clinical isolates of *Bacillus subtilis*, *Micrococcus luteus*, *Staphylococcus aureus*, *Klebsiella pneumoniae*, and *Enterobacter aerogenes* were sensitive to all the oils, while those of *Pseudomonas aeruginosa*, *Escherichia coli*, and *Proteus vulgaris* were resistant to the Shathari, Najdi, and Hoojri oils, respectively. The resistance of some of the Gram-negative bacteria to some of the oils could be due to the more hydrophilic outer membrane containing lipopolysaccharide. Small hydrophilic molecules are able to pass the outer membrane through porin channels, while the outer membrane acts as a penetration barrier for macromolecules and hydrophobic compounds. But the outer membrane is not completely impermeable to hydrophobic molecules; some of them can slowly pass through the porins. Hence, passing through the outer membrane contributes to the bactericidal activity of a compound. This could be the possible explanation for the sensitivity of some Gram-negative bacteria to the different luban oils [34].

Recently Abdoul-latif et al. [49] reported the antibacterial activity of essential oils of *B. sacra* and *B. papyrifera*. The best zone of inhibition of essential oil of *B. sacra* for bacteria was obtained for *Enterococcus faecalis* (37 mm), *Shigella dysenteria* (37 mm), *Salmonella enterica* (35 mm), *Bacillus cereus* (34 mm), and *Listeria innocua* (34 mm). Similarly best zone of inhibition of essential oil of *B. papyrifera* for bacteria was obtained for *Salmonella enterica* (40 mm), *Bacillus cereus* (39 mm), *Enterococcus faecalis* (39 mm), *Shigella dysenteria* (31 mm), and *Staphylococcus camorum* (30 mm). Interestingly essential oils of *B. sacra* and *B*. *papyrifera* present an antimicrobial activity stronger than the tetracycline.

### 3.4. Anticancer Activity

Frankincense oil-induced cell viability was investigated for essential oils of *B. carterii* in human bladder cancer J82 cells and immortalized normal bladder urothelial UROtsa cells [50]. The results showed that within a range of concentrations, frankincense oil suppressed cell viability in bladder transitional carcinoma J82 cells but not UROtsa cells. Comprehensive gene expression analysis confirmed that frankincense oil activated genes that were responsible for cell cycle arrest, cell growth suppression, and apoptosis in J82 cells. However, frankincense oil-induced cell death in J82 cells did not result in DNA fragmentation, a hallmark of apoptosis. Therefore, frankincense oil appeared to distinguish cancerous from normal bladder cells and suppress cancer cell viability. Microarray and bioinformatics analysis proposed multiple pathways that could be activated by frankincense oil to induce bladder cancer cell death [50]. 

Recently, Suhail et al. [51] showed that *B. sacra* essential oil suppressed important malignant features of tumor cells, such as invasion and multicellular tumor spheroid growth. Tumor cell plasticity enables highly malignant tumor cells to express endothelial cell-specific markers and form vessel-like network structures on basement membranes. The in vitro Matrigel-based tumor invasion model has been shown to correlate with in vivo metastatic potential [52]. This in vitro model has been used to study mechanisms of cancer aggressive behavior, metastasis, and poor prognosis [53], and it has been used as a tool to screen therapeutic agents for antimetastatic activity [54, 55]. MDA-MB-231 cells grown on Matrigel are more resistant to essential oil-suppressed cell viability than cells grown on tissue culture plates. This difference may result from the protective effects of the Matrigel basement membrane matrix enriched with various growth factors. In addition, cancer cells can form multicellular spheroid aggregates, which afford protection for cancer cells against some chemotherapeutic agents [56]. 

Multicellular tumor spheroids in culture have been used as an in vitro model for screening and testing anticancer drugs [57]. Similar to results from cytotoxicity and apoptosis, *B. sacra* essential oil obtained at 100°C in hydrodistillation is more potent than essential oil obtained at 78°C in disruption of cellular networks on Matrigel and spheroids. More importantly, observations obtained in the above-described experimental models were consistent with clinical responses in human cancer cases. These results suggested that *B. sacra* essential oil might represent an effective therapeutic agent for treating invasive breast cancer. 

Aberrant activations of Akt and ERK1/2 MAPK signaling molecules have been identified in various cancers including breast cancer, and activations of Akt and ERK1/2 have been suggested as independent cancer prognostic markers. The Akt pathway has been found to be activated in early stages of breast cancer development [58], and activation of Akt signaling protects breast cancer cells from tamoxifen-induced apoptosis in vitro and confers poor prognosis in cancer patients [59, 60]. Activation of ERK1/2 has also been shown to be associated with the development of tamoxifen resistance and patient survival [61, 62]. Both Akt and ERK1/2 have been proposed as molecular targets for treating breast cancer, particularly in antiestrogen-resistant states [63, 64]. Targeting Akt signaling by inhibiting mTRO signaling has been shown to restore cancer responses to chemotherapy drugs [65, 66], and inhibition of both epidermal growth factor receptor (EGFR)/HER2 and MAPK signaling has been shown to result in growth inhibition and apoptosis of EGFR-expressing breast cancer cells [67]. Studies have shown that boswellic acids and AKBA activate the PI3 K/Akt pathway in human colon cancer HT29 cells [68]. Suhail et al. [51] demonstrated that *B. sacra* essential oil suppressed Akt and ERK1/2 activation in human breast cancer cell lines, except MDA-MB-231. The differences observed between boswellic acids and *B. sacra* essential oil may result from different tested tumor cell types or components other than boswellic acids present in the essential oil [51]. 

### 3.5. Antibiofilm Activity

Schillaci et al. [47] evaluated anti-biofilm activity of the commercially available essential oils from *B. papyrifera* against the preformed 24 h old biofilms of two bacterial strains: *Staphylococcus epidermidis* DSM 3269 and *Staphylococcus aureus* ATCC 29213. Interestingly, the anti-biofilm activity exhibited at the lowest concentrations of 13.6 *μ*g/mL (1.5% v/v) and 6.8 *μ*g/mL (0.75% v/v) was below that of the MIC concentration of 22.6 *μ*g/mL (2.6% v/v), as determined against planktonic forms of both bacterial strains. These data were curious, considering that staphylococcal biofilms are usually resistant to conventional antibiotics at concentrations up to 1000 times the MIC. 

## 4. Conclusion

None of the volatiles identified in the different studies have, according to our knowledge, ever been attributed to the specific smell of frankincense. It is interesting to note, however, that an olibanum-like odour has been reported elsewhere for a substance found in orange oil residue [21] which was identified as cis-iso-cascarilla acid. Nevertheless, this compound has not been reported as a constituent of frankincense in the literature discussed in this paper. 

Furthermore, it remains unanswered whether there are substances with frankincense-specific odour qualities, or whether the characteristic smell of frankincense is due to a specific blend of dorants, as often observed in other food or plant aromas. Further research is therefore necessary to elucidate the specific contributors to the aroma profile of frankincense and frankincense pyrolysate. The essential oils of *Boswellia* plants showed different activities which is summarized in Table 3.

## Figures and Tables

**Table 1:** Essential oil of *Boswellia* spp.

Number	Compound
1	5,5-Dimethyl-1-vinylbicyclo-[2.1.1]-hexane
2	Anethol
3	Benzyl tiglate
4	*trans*-*α*-Bergamotene
5	Bornyl acetate
6	*β*-Bourbonene
7	Cadinene
8	*γ*-Cadinene
9	Camphene
10	Camphor
11	*m*-Camphorene
12	*p-*Camphorene
13	Carene-3
14	(*E*)-*β*-Caryophyllene
15	Cembrene A
16	Cembrenol
17	1,8 Cineol
18	Citronellol
19	*α*-Copaene
20	*β*-Copaene
21	*p*-Cymene
22	*m-*Cymene
23	Elemol
24	Elemicine
25	*epi*-Cubenol
26	Estragol
27	Eudesmol
28	10-*epi*-*γ*-Eudesmol
29	Fenchone
30	Geraniol
31	Germacrene D
32	Humulene epoxide
33	Isoincensole
34	Isomenthone
35	Kessane
36	Limonene
37	Linalool
38	Linalyl acetate
39	Menthone
40	Methylchavicol
41	Methylisoeugenol
42	Methyleugenol
43	*γ*-Muurolene
44	Myrcene
45	Neocembrene A
46	Nerolidol
47	*cis*-*β*-ocimene
48	*(Z)-*Ocimene
49	*(E)-β* *-*Ocimene
50	Perillene
51	*α*-Phellandrene
52	*β*-Phellandrene
53	*α*-Pinene
54	*β*-Pinene
55	*trans*-Pinocarveol
56	Sabinene
57	*cis*-Sabinol
58	Terpinin-4-ol
59	Terpinen-4-ol
60	Terpinolene
61	*α*-Terpineol
62	*α*-Terpinene
63	*α*-Terpinene
64	*γ*-Terpinene
65	Terpinyl acetate
66	Terpinyl isobutyrate
67	Tetrahydrolinalool
68	*α*-Thujene
69	*α*-Thujone
70	*β*-Thujone
71	Tricyclene
72	Undecenol
73	*trans*-Verbenol
74	*β*-Ylangene
75	Zingiberene
76	Abieta-8,12-diene
77	*α*-Amorphene
78	*allo*aromadendrene
79	Benzyl benzoate
80	Beyerene
81	Bisabolene
82	Isopentyl-2-methylbutanoate
83	*cis*-Calamenene
84	*α*-Cadinene
85	*τ*-Cadinol
86	2-Carene
87	Campholenealdehyde
88	Caryophyllene oxide
89	*cis*-Carveol
90	(+) *trans*-Carveol
91	Carvone
92	*α*-Cedrene
93	Cedrol
94	Cembra-1,3,7,11-tetraene
95	Cembra-3,7,11,15-tetraene
96	Cembrene
97	Cembrene C
98	Citronellyl acetate
99	*α*-Cubebene
100	*β*-Cubebene
101	*o*-Cymene
102	Chrysanthenone
103	1,4-Cyclohexadiene
104	*p*-Cymen-8-ol
105	Decanol
106	Decyl acetate
107	2,6-Dimethoxytoluene
108	3,5-Dimethoxytoluene
109	Duva-3,9,13-trien-1,5*α*-diol
110	Duva-4,8,13-trien-1a,3*α*-diol
111	Duva-3,9,13-trien-1,5*α*-diol-1-acetate
112	Duva-3,9,13-triene-1*α*-ol-5,8-oxide-1-acetate
113	*β*-Elemene
114	Farnesyl acetate
115	Geranyl acetate
116	*α*-Gurjunene
117	Hedycariol
118	1,3,6-Trimethylencycloheptane
119	1-Hexanol
120	Hexyl acetate
121	Hexyl hexanoate
122	*α*-Humulene
123	Incensole
124	Incensole acetate
125	Isodurene
126	Isocembrene
127	Isophyllocladene (kaur-15-ene)
128	Kaurene
129	Ledol
130	Maaliane
131	*p*-Mentha-1,5-dien-8-ol
132	*o*-Methyl anisole
133	*α*-Muurolene
134	*α*-Muurolol
135	Myrtenal
136	Naphthalene
137	Naphthalene 1,2,3,4,4a,7-hexahydro-1,6-dimethyl-4-(1-methylethyl
138	Neryl acetate
139	*cis*-Nerolidol
140	(*S*)-*trans*-Nerolidol
141	(*E*)-Nerolidol
142	1-Octanol
143	*n*-Octanol
144	Octanol acetate
145	Octyl acetate
146	Octyl formate
147	*allo*-Ocimene
148	Phenanthrene-7-ethenyl-9,10,10a-dodeca-hydro-1-1-4a- 7-tetramethyl
149	*α*-Phellandrene epoxide
150	Phyllocladene
151	*α*-Pinene-epoxide
152	1-*β*-Pinene
153	2-*β*-Pinene
154	Isopinocampheol
155	Piperitone
156	Pyrimidine
157	Sabinyl acetate
158	Sandaracopimara-8(14)-15-diene
159	Sclarene
160	*α*-Selinene
161	*β*-Selinene
162	*δ*-Selinene
163	*trans*-Terpine
164	4-Terpineol
165	Terpinolene
166	Isoterpinolene
167	2,4(10)-Thujadiene
168	Thujopsene
169	Thunbergol
170	Isomyl-valerate
171	Verticilla-4(20),7,11-triene
172	Verbenone
173	*cis*-Verbenol
174	Verticiol
175	Viridiflorol
176	Benzene, 1methoxy-2-methyl
177	*endo*-Borneol
178	*γ*-Campholene aldehyde
179	*α*-Campholene aldehyde
180	Cara-2,4-diene
181	Carvacrol
182	Carvotanacetone
183	*trans-*Dihydrocarvone
184	Cumin alcohol
185	*m*-Cymene-8-ol
186	*p*-Cymene-9-ol
187	*p*-Cymenene
188	Dodecanol
189	Eucalyptol
190	Eucarvone
191	Isopropyl benzaldehyde
192	Isopropyl benzalcohol
193	*cis-*1,2-Limonene epoxide
194	8,9-Limonene epoxide II
195	8,9-Limonene-epoxide I
196	*trans-*1,2-Limonene epoxide
197	*cis*-Linalool oxide
198	*trans*-Linalool oxide
199	*p*-Mentha-1,5-diene-7-ol
200	*p*-Mentha-1,8-diene-4-ol
201	*cis*-*p*-Menth-2-en-1-ol
202	*cis*-*p*-Mentha-1(7),8-diene-2-ol
203	*cis*-*p*-Mentha-2,8-diene-1-ol
204	*trans*-*p*-Menth-2-en-1-ol
205	*trans*-*p*-Mentha-1(7),8-diene-2-ol
206	*trans*-*p*-Mentha-2,8-diene-1-ol
207	2,4(8)-*p*-Menthadiene
208	*p*-Mentha-6,8-dien-2-one
209	*p*-Methylanisole
210	Myrtenol
211	Nerol
212	*trans*-Ocimene
213	(*E*)-*β*-Ocimene epoxide
214	*α*-Phellandrene-dimer
215	*α*-Phellandrene-8-ol
216	*α*-Pinene oxide
217	Pinocamphone
218	Pinocarvone
219	Piperitenone
220	Isopiperitenone
221	*trans*-Piperitol
222	*α*-Terpineol
223	Sabina ketone
224	*cis*-Sabinene hydrate
225	*trans*-Sabinene hydrate
226	*trans-*Sabinol
227	2,5-Dimethylstyrene
228	*cis*-1,2-Epoxy-terpin-4-ol
229	Thuj-3-en-10-al
230	Thujanol
231	Thunbergene
232	Thymol
233	Umbellulone
234	Verticellol
235	5,5-Dimethyl-1-vinylbicyclo-[2.1.1]-hexane
236	*p*-Anisaldehyde
237	Aromadendrene
238	Benzyl tigilate
239	*p-*Camphorene
240	Isocaryophyllene
241	Cumaldehyde
242	Cyclosativene
243	*γ*-Eudesmol
244	Guaioxide
245	5-Guaiene-11-ol
246	Isogermacrene D
247	4-Methylene-1-(1-methylethyl)-bicyclo[3.1.0]hex-2-ene
248	2-Methyl-5-(1-methylethyl)-1,3-cyclohexadiene monoepoxide
249	*n*-Pentadecan
250	Perilla alcohol
251	Perillol
252	Thujol
253	*m*-Thymol
254	*α*-Ylangene
255	*γ*-Campholene aldehyde
256	*n*-Decanoic acid
257	*β*-Eudesmene
258	*β*-Cyclogeranylacetate
259	*n*-Hexanoic acid
260	Hexylcaprylate
261	Incensyl acetate
262	Incensole oxide
263	Incensole oxide acetate
264	Lauric acid
265	*p-*Methylacetophenone
266	*p*-Methyleugenol
267	*β*-Myrcene
268	*n*-Nonanoic acid
269	*n*-Octanoic acid
270	3,4-Dimethoxystyrene
271	*α*-Cadinol
272	1,Hydroxy-1,7-dimethyl-4-isopropyl-2,7-cyclodecadiene
273	1,5,5,8-Tetramethyl-12-oxabicyclo-[9.1.0]-dodeca-3,7-diene
274	1-Methyl-4-(1-methylethenyl)-1,2-cyclohexanediol
275	*trans-p*-Mentha-2,8-dienol
276	1,2,3,4,6,8a-hexahydro-1-isopropyl-4,7-dimethyl- naphthalene
277	2-Isopropenyl-4a,8-dimethyl-1,2,3,4,4a,5,6,8a-ctahydronaphthalene
278	3,5-Dimethoxytoluene
279	(*Z*)-*α*-Hydroxymanool
280	Hydroxy-manool
281	Methyl linoleate
282	1-Acetyl-4-isopropenylcyclopentene
283	2,4-Dimethylacetophenone
284	*α*-Amyrenone
285	*β*-Amyrenone
286	10-Hydroxy-4-cadinen-3-one
287	2-Hydroxy-1,4-cineole
288	Cryptone
289	Eucarvone
290	Isopropylidencyclohexane
291	1,2,4-Trihydroxy-*p*-menthane
292	Δ^4^-*p*-Menthen-2-one
293	5-Hydroxy-*p*-menth-6-en-2-one
294	Myrtenoic acid
295	Nopinone
296	3,6,6,-Trimethyl-norpinan-2-one
297	*o*-Methylacetophenone
298	Perillaaldehyde
299	Phellandra
300	Pinocamphone/isopinocamphone
301	Thujone
302	24-Noroleana-3,12-diene
303	24-Noroleana-3,9(11),12-triene
304	24-Norursa-3,12-diene
305	24-Norursa-3,9(11),12-triene
306	24-Norursa-3.12-dien-11-one
307	*α*-Amyrine
308	*epi*-*α*-Amyrine
309	*β*-Amyrine
310	Lupeol
311	Terpinenyl acetate
312	1,5-Isopropyl-2-methylbicyclo[3.1.0]hex-3-en-2-ol
313	*α*-Campholenal
314	(3*E*,5*E*)-2,6-Dimethyl-1,3,5,7-octatetraene
315	(*E*)-2,3-Epoxycarene
316	3,4-Dimethylstyrene
317	1-(2,4-Dimethylphenyl)ethanol
318	4-Methylbenzoic acid
319	*p*-Menth-1(7)-en-2-one
320	Caryophyllene
321	Methylcycloundecanecarboxylate
322	Nonanoic acid
323	Hexadecanoic acid
324	1,4-Cineol
325	Sabinene hydrate
326	Methyl-*trans*-2-*cis*-4-decadienoate
327	2-Hydroxy-5-methoxy-acetophenone
328	(*E*)-*β*-Farnesene
329	2-Dodecenoic acid methyl ester
330	Calacorene
331	*n*-Dodecanoic acid
332	**α*-*Guaiol
333	Caryophylla-3(15),7(14)-dien-6-ol
334	Cadalene
335	Eudesma-4(15),7-dien-1*β*-ol
336	*n*-Heptadecane
337	*n*-Tetradecanoic acid
338	*n-*Octadecane
339	Galaxolide
340	Manool

**Table 2:** Percentages of major compounds in the essential oils of reported *Boswellia* species.

*Boswellia* specie	Method of obtaining resin	Predominant compound(s)	Percentage (%)	Literature
*B. serrata *	Obatined from Willy Benecke GmbH (Hamburg, Germany)	Myrcene	38	[16]
*B. serrata *	NA	*α*-Thujene	22.7–47.4	[22]
*B. serrata *	NA	*α*-Thujene	29.3	[24]
*B. serrata *	NA	*α*-Thujene	61.36	[23]
*B. carteri *	Purchased from the local market of herbs and spices in Egypt	Duva-3,9,13-triene-1a-ol-5,8-oxide-1-acetate	21.4	[20]
*B. sacra *	Botanically certified oleogum resin	*E*-*β*-Ocimene	32.3	[25]
*B. carteri/sacra *	NM	Octanol acetate	45.2	[26]
*B. carteri *	Authentic sample from Ethiopia certified for its authenticity from the Agricultural Department of the Ethiopian government	Octyl acetate	39.3	[16]
*B. rivae *	NA	Limonene	28.0	[24]
*B. rivae *	Authentic sample from Ethiopia	*α*-Pinene	16.7	[16]
*B. rivae *	NA	*α*-Pinene	13.3	[24]
*B. rivae *	NA	Octanol	17.8	[24]
*B. neglecta *	NA	*α*-Pinene	16.7	[27]
*B. neglecta *	Authentic sample from Ethiopia	*α*-Pinene	21.3	[16]
*B. papyrifera *	NA	Octyl acetate	63.5	[24]
*B. papyrifera *	NA	Octyl acetate	56.0	[36]
*B. pirottae *	NA	*Trans*-Verbenol	15.5	[27]
*B. pirottae *	NA	Terpinen-4-ol	14.6	[27]
*B. frereana *	Willy Benecke GmbH (Hamburg, Germany)	*α*-Pinene	38.0	[16]

NA: not available.

**Table 3:** Biological activities of essential oils of *Boswellia* genus.

Plants	Biological activities of essential oils of *Boswellia* planta				
	Antioxidant	AchEI inhibition	Antimycrobial	Anticancer	Antibiofilm
*B. socotrana *	IC_50_ 121.4 *μ*g/mL,	59.3%	Moderate activity	NK	NK
*B. elongata *	IC_50_ 211.2 *μ*g/mL	29.6	Moderate activity	NK	NK
*B. ameero *	IC_50_ 175.2 *μ*g/mL	41.5	NK	Good activity	NK
*B. carteri *	NK^a^	NK	Moderate activity		NK
*B. neglecta *	NK	NK	Moderate activity		NK
*B. sacra *	NK	NK	Good activity	Good activity	NK
*B. thurifera *	NK	NK	Moderate activity		NK
*B. frereana *	NK	NK	Moderate activity		NK
*B. dioscorides *	NK	NK	Moderate activity		NK
*B. rivae *	NK	NK	Good activity		NK
*B. papyrifera *	NK	NK	Good activity		Good activity

^a^NK: not known.
